This article has been retracted.

# TIPE2 suppresses progression and tumorigenesis of esophageal carcinoma via inhibition of the Wnt/β-catenin pathway

**DOI:** 10.1186/s12967-018-1383-0

**Published:** 2018-01-17

**Authors:** Linan Zhu, Xudong Zhang, Xiaorui Fu, Zhaoming Li, Zhenchang Sun, Jingjing Wu, Xinhua Wang, Feng Wang, Xiangke Li, Songtao Niu, Mengjie Ding, Zhenzhen Yang, Wanqiu Yang, Meifeng Yin, Lei Zhang, Mingzhi Zhang

**Affiliations:** Department of Oncology, The First Affiliated Hospital of Zhengzhou University, Νo. 1 Jianshe East Road, Zhengzhou, 450052 Henan People’s Republic of China

**Keywords:** Esophageal carcinoma, TIPE2, Proliferation, Tumorigenesis, Wnt/β-catenin pathway

## Abstract

**Background:**

Esophageal carcinoma is the eighth prevalent malignancy and ranks the sixth in carcinoma-related death worldwide. Tumor necrosis factor-α-induced protein-8 like-2 (TIPE2) has been identified as a tumor suppressor in multiple carcinomas. However, its roles and molecular mechanisms underlying esophageal carcinoma progression are still undefined till now.

**Methods:**

RT-qPCR assay was employed to detect the expression of TIPE2 mRNA. TIPE2 protein expression was measured by using western blot assay. Ad-V and Ad-TIPE2 adenoviruses were constructed to overexpress TIPE2. The effects of TIPE2 overexpression on cell proliferation, invasion and apoptosis were assessed by MTT and Edu incorporation assays, transwell invasion assay and flow cytometry analysis, respectively. The effect of TIPE2 overexpression on xenograft tumor growth was determined by measuring tumor volume and weight, together with immunohistochemistry assay. The effect of TIPE2 overexpression on the Wnt/β-catenin signaling pathway was evaluated by detecting the protein levels of β-catenin, c-Myc and cyclinD1 in EC9076 cells and xenograft tumors of esophageal carcinoma.

**Results:**

TIPE2 expression was downregulated in esophageal carcinoma tissues and cells. Adenovirus-mediated TIPE2 overexpression suppressed cell proliferation and invasion, and induced apoptosis in esophageal carcinoma cells. Enforced expression of TIPE2 inhibited tumor growth in vivo, as evidenced by the reduced tumor volume, tumor weight and proliferating cell nuclear antigen expression. Overexpression of TIPE2 inhibited the Wnt/β-catenin signaling pathway in esophageal carcinoma in vitro and in vivo.

**Conclusions:**

These results suggest that TIPE2 suppressed progression and tumorigenesis of esophageal carcinoma via inhibition of the Wnt/β-catenin pathway.

## Background

Esophageal carcinoma, a malignant tumor of gastrointestinal tract, contains two major subtypes of adenocarcinoma and squamous cell carcinoma [1]. Esophageal carcinoma is the eighth prevalent tumor in all malignancies and ranks the sixth in cancer-related death worldwide [2]. In 2016, there was an estimated 16,940 new cases (1% of all new carcinoma cases) and 15,690 deaths (2.6% of all carcinoma-associated deaths) of esophageal carcinoma occurred in USA [3]. Although much progress has been made in the diagnose and therapy of esophageal carcinoma, its 5-year survival rate is still unsatisfactory [3, 4]. Therefore, further exploring the molecular basis underlying esophageal carcinoma tumorigenesis and figuring out more effective therapeutic strategies are imperative.

Human tumor necrosis factor-α-induced protein-8 like-2 (TIPE2, TNFAIP8L2), located on chromosome 1q21.2–1q21.3, shared 94% identical amino acid sequence with murine TIPE2 [5]. TIPE2 is a vital negative regulator of immune and inflammation homeostasis, which is closely associated with the development and progression of cancer [5–8]. Recent studies showed that TIPE2 was downregulated and acted as a tumor suppressor in non-small cell lung cancer [9], glioma [10], prostate carcinoma [11] and gastric carcinoma [12, 13]. However, its roles and molecular mechanisms underlying esophageal carcinoma progression are still undefined till now.

In the present study, we firstly demonstrated that TIPE2 expression was downregulated in esophageal carcinoma tissues and cells. Functional and mechanistic analyses revealed that TIPE2 overexpression repressed the progression of esophageal carcinoma in vitro and in vivo by inhibiting the Wnt/β-catenin pathway.

## Methods

### Tissues samples

Tumor tissue specimens and the corresponding adjacent normal tissues were obtained from 29 patients diagnosed with esophageal carcinoma (19 males, 10 females; 50–70 years old) at the First Affiliated Hospital of Zhengzhou University between August 2014 and January 2016. Before surgery resection, none of the patients had received any radiotherapy or chemotherapy. The surgically resected specimens were immediately snap-frozen in liquid nitrogen and stored at − 80 °C for the subsequent assays. Our study was performed with the approval of Ethics Committee of the First Affiliated Hospital of Zhengzhou University and written informed consent was obtained from every patients.

### Cell lines and culture

Human esophageal carcinoma cell lines (EC9076, KYSE410, KYSE150, TE-1 and EC109) and human normal esophageal epithelial cells HEEC were purchased from Cell Bank of Chinese Academy of Science (Shanghai, China). These cells were grown in RPMI-1640 medium (Hyclone, Logan, UT, USA) containing 10% heat-inactivated fetal bovine serum (FBS; Invitrogen, Carlsbad, CA, USA) and 1% penicillin/streptomycin (Invitrogen; Thermo Fisher Scientific, Inc., Waltham, MA, USA) at 37 °C in a humidified chamber with 5% CO_2_.

### Adenovirus preparation and transduction

The full length coding sequences of TIPE2 were amplified and constructed into pAdTrack-CMV shuttle plasmid with the name of pAdTrack-CMV-TIPE2, followed by the recombination of pAdTrack-CMV-TIPE2 and pAdEasy-1 backbone vector to generate pAd-TIPE2 recombination plasmids. Meanwhile, the control pAd-V recombination plasmid was also generated using the same method. After transfection for 8–10 days, pAd-V and pAd-TIPE recombination plasmids were transfected into HEK 293 cells using Lipofectamine 2000 (Invitrogen) to generate Ad-V and Ad-TIPE2 adenovirus, respectively. The titer of adenovirus was determined using plaque formation assays.

After EC109 and EC9706 cells seeded in 24-well plates were grown to 80% confluence, they were infected with recombinant adenovirus Ad-V and Ad-TIPE2 at multiplicity of infection (MOI) of 50.

### Reverse transcription-quantitative polymerase chain reaction (RT-qPCR) assay

Total RNA was extracted from tissues and cells using the Trizol reagent (Invitrogen) following the instructions of manufacturer. Then 1 μg RNA was reversely transcribed into cDNA using M-MLV reverse transcriptase (Invitrogen) and random primers. Fast SYBR Green Master Mix (Applied Biosystems, Foster City, CA, USA) was used to detect expression of TIPE2 mRNA on the Applied Biosystems 7500 Fast Real-Time PCR System (Applied Biosystems), with β-actin as an endogenous control. The primers sequences of TIPE2 and β-actin were listed as follows: TIPE2, 5′-ACT GAG TAA GAT GGC GGG TCG-3′ (forward) and 5′-TTC TGG CGA AAG CGG GTA G-3′ (reverse); β-actin, 5′-AAA TCG TGC GTG ACA TCA AAG A-3′ (forward) and 5′-GGC CAT CTC CTG CTC GAA-3′ (reverse).

### Western blot assay

Total proteins were extracted from cells and tissues using RIPA buffer (Beyotime, Shanghai, China) containing protease inhibitor cocktail (Roche Diagnostics, Basel, Switzerland) and quantified using a Pierce™ BCA protein assay kit (Invitrogen; Thermo Scientific). Then equal amount of proteins (50 µg) were separated using 10% sodium dodecyl sulphate–polyacrylamide gel electrophoresis (SDS-PAGE) and transferred onto nitrocellulose filter membrane (NC membrane; Millipore, Billerica, MA, USA). Next, the membranes were blocked in 5% skim milk for 1 h at room temperature and probed with primary antibodies against TIPE2 (ab110389, 1:1000, Abcam, Cambridge, MA, USA), β-actin (ab8227, 1:5000, Abcam), β-catenin (ab32572, 1:5000, Abcam), c-Myc (ab32072, 1:1000, Abcam), and cyclinD1 (ab134175, 1:1000, Abcam) overnight at 4 °C, followed by the incubation with horseradish peroxidase (HRP)-conjugated goat-anti rabbit second antibodies (ab6721, 1:1000, Abcam) for 1 h at room temperature. At last, specific protein signal was visualized using a ECL western blotting substrate (Promega, Madison, WI, USA) and quantified by A Image J software (National Institutes of Health, Bethesda, Maryland, USA).

### Methylthiazolyldiphenyl-tetrazolium bromide (MTT) assay

EC9076 and EC109 cells (10^4^/well) were seeded into 96-well plates and incubated overnight in a humidified atmosphere with 5% CO_2_ at 37 °C. Then, the cells were infected with Ad-V or Ad-TIPE adenovirus at a dose of 50 multiplicity of infection (MOI). At the indicated time points (day 0, 1, 2, 3) following infection, 20 μl MTT solution (5 mg/ml, Sigma-Aldrich, St. Louris, MO, USA) was added into each well. After incubation for another 4 h at 37 °C, the medium was discarded and 150 μl dimethyl sulfoxide (DMSO, Sigma-Aldrich) was carefully added into each well to dissolve formed formazan precipitates. Optical density (OD) values were measured at the wavelength of 490 nm on a microplate reader (Molecular Devices, Sunnyvale, CA, USA).

### 5-Ethynyl-2′-deoxyuridine (EdU) cell proliferation assay

Baseclick EdU-Click 488 kit (Sigma-Aldrich) was used to detect cell proliferation. Briefly, EC9076 and EC109 cells were seeded on cover slips and then infected with Ad-V or Ad-TIPE2 adenovirus for 3 days. Next, the cells were maintained for 3 h in serum-medium containing 50 μM final concentration of Edu, followed by fixation with 4% formaldehyde in PBS for 15 min and permeabilization using 0.5% Triton^®^ X-100 in PBS for 20 min at room temperature. Then, permeabilization solution was removed and 500 μl of the reaction cocktail was added to each well with a coverslip for 30 min in the dark. Subsequently, cells were processed by 0.1 μg/ml of DAPI for 10 min to stain cell nucleus in the dark. At last, cells were imaged with a confocal laser-scanning microscope (LSCM, Leica Microsystems, Solms, Germany). The relative proliferation rate was calculated following the formula: relative proliferation rate = Edu-incorporated cell numbers/DAPI-stained cell numbers. The relative proliferation rate was normalized by Ad-V-infected group.

### Transwell invasion assay

Cell invasion capability was assessed using an invasion chamber (BD Bioscience, San Diego, CA, USA) with 8 μm pore-size membrane (BD Bioscience). Briefly, EC9076 and EC109 cells (10^5^/well) infected with Ad-V or Ad-TIPE2 were resuspended in serum-free RPMI-1640 medium (100 μl) and seeded into the upper chamber pre-coated with 40 µl Matrigel (BD Biosciences), while the lower chamber was filled with 700 μl RPMI-1640 medium containing 10% FBS. Following a 48 h incubation at 37 °C, the cells on the upper sides of membranes were removed by a sterile cotton swab. The cells on the bottom sides of membranes were fixed with methanol for 30 min, stained with 0.1% crystal violet for 20 min, and counted in 6 randomly selected fields using the inverted microscope (Nikon Eclipse TE300, Tokyo, Japan) at ×200 magnification.

### Flow cytometry for apoptosis detection

Cell apoptosis rates were determined using a Annexin V-FITC/propidium iodide (PI) apoptosis detection kit (Nanjing Kaiji Biotechnology Development Co., Ltd., Nanjing, China) following the protocols of manufacturer. Briefly, EC9076 and EC109 cells were infected with Ad-V or Ad-TIPE2 adenovirus for 3 days. Then the cells were collected and resuspended in 500 μl 1 × Binding Buffer at a concentration of 1 × 10^6^ cells/ml, followed by the addition of 5 μl Annexin V-FITC and 5 μl PI. Then the treated cells were incubated for 5 min in the dark at room temperature. Finally, a FACS Calibur Flow Cytometer (Beckman Coulter, Atlanta, GA, USA) was used to measure the apoptosis rate of cells.

### In vivo experiment

BALB/c nude mice (6–7 weeks old, male) were obtained from Chinese Academy of Science (Shanghai, China) and grown in specific pathogen-free conditions. All animal studies were performed according to the Guide for the Care and Use of Laboratory Animals of Zhengzhou University. To explore the effect of TIPE2 overexpression on tumor growth in vivo, EC9706 cells infected with Ad-V or Ad-TIPE2 at a concentration of 1 × 10^7^ cells/ml were injected subcutaneously into the flank region of nude mice. Tumor volume was measured every 3 days for 9 times with a caliper following the formula of 0.5 × length × width^2^. At day 24 after injection, the tumors of all mice were obtained, weighted and fixed in formalin for the following assays.

### Immunohistochemical (IHC) assay

Surgically excised xenograft tumor specimens were fixed with 10% formalin and embedded in paraffin, followed by deparaffinization, rehydration, endogenous peroxidase blocking, and antigen retrieval. Then the specimens were blocked with 1% bovine serum albumin (BSA) for 10 min at room temperature and incubated with proliferating cell nuclear antigen (PCNA) antibody (ab18197, 1:1000, Abcam) overnight at 4 °C, followed by incubation with HRP-labeled secondary antibody (ab6721, 1:1000, Abcam) for 1 h at 37 °C. Next, DAB Peroxidase Substrate kit (General bioscience, Brisbane, California, USA) was used to visualize the immunoreactivity. For hematoxylin–eosin (H&E) staining, tissues were counterstained with hematoxylin–eosin and then photographed using a microscope (Nikon Eclipse TE300, Tokyo, Japan). Blue stands for cell nucleus and red or pink is an indicator of cytoplasm in H&E staining. Positive PCNA displays brown in IHC.

### Statistical analysis

All data were obtained from three independent experiments and presented as mean ± standard deviation (mean ± SD). Student’s *t*-test or one-way ANOVA was employed to explore the difference of data in different groups. Differences were statistically significant when *P* < 0.05.

## Results

### TIPE2 expression was downregulated in esophageal carcinoma tissues and cells

Firstly, RT-qPCR assay was performed to detect TIPE2 expression in 29 pairs of esophageal carcinoma tissues and adjacent normal tissues. As shown in Fig. 1a, TIPE2 mRNA expression was notably downregulated in esophageal carcinoma tissues compared with the corresponding adjacent normal tissues. Moreover, the protein levels of TIPE2 were significantly decreased in 29 esophageal carcinoma tissues compared with adjacent normal tissues (Fig. 1b). Furthermore, western blot assay manifested that TIPE2 was also distinctly downregulated in esophageal carcinoma cell lines (KYSE410, EC9706, KYSE150, TE-1, and EC109) than that in normal human esophageal epithelial cells (HEEC) (Fig. 1c). These findings imply a possible role for TIPE2 in the pathogenesis of esophageal carcinoma.

**Fig. 1:** TIPE2 expression was downregulated in esophageal carcinoma tissues and cells. **a** RT-qPCR assay was used to detect TIPE2 mRNA expression in 29 pairs of esophageal carcinoma tissues and adjacent normal tissues, with β-actin as an endogenous control. **b** The overall expression of TIPE2 protein in 29 pairs of esophageal carcinoma tissues and adjacent normal tissues was measured using western blot and normalized to β-actin expression. **c** TIPE2 protein level in esophageal carcinoma cell lines (KYSE410, EC9706, KYSE150, TE-1, and EC109) and normal human esophageal epithelial cells (HEEC), *P < 0.05

### TIPE2 overexpression suppressed the proliferation of esophageal carcinoma cells

To determine the effect of TIPE2 overexpression on the progression of esophageal carcinoma, the coding sequence of TIPE2 was cloned into the recombinant adenovirus vectors to generate Ad-TIPE2 adenovirus, followed by adenovirus infection into EC9706 and EC109 cells. The following western blot assay further demonstrated that TIPE2 protein level was significantly increased in Ad-TIPE2-infected EC9706 (Fig. 2a) and EC109 cells (Fig. 2b) compared with Ad-V-infected cells. Then, the effect of TIPE2 overexpression on the proliferation of EC9706 and EC109 cells was further investigated. MTT assay revealed that adenovirus-mediated TIPE2 overexpression markedly suppressed proliferation of EC9706 (Fig. 2c) and EC109 (Fig. 2d) cells at day 2 and 3 after infection compared with Ad-V control group. Moreover, EdU cell proliferation assay further demonstrated that adenovirus-mediated TIPE2 overexpression resulted in an obvious decrease of EdU incorporated cell numbers in EC9706 (Fig. 2e) and EC109 (Fig. 2f) cells compared with Ad-V-infected cells. EdU quantification results further revealed that the proliferation rates of cells were remarkably reduced in Ad-TIPE2-infected EC9706 (Fig. 2g) and EC109 (Fig. 2h) cells than that in Ad-V-infected cells. Collectively, these results demonstrated that TIPE2 overexpression suppressed the proliferation of esophageal carcinoma cells.

**Fig. 2:** TIPE2 overexpression suppressed the proliferation of esophageal carcinoma cells. TIPE2 protein level in PBS-treated, Ad-V- or Ad-TIPE2-infected EC9706 (**a**) and EC109 (**b**) cells were measured using western blot assay after treatment for 3 days. MTT assay was performed to detect the proliferation of EC9706 (**c**) and EC109 (**d**) cells at the indicated time points (0, 1, 2, 3 days) after infection with Ad-V or Ad-TIPE2. Representative images of EdU incorporation in Ad-V- or Ad-TIPE2-infected EC9706 (**e**) and EC109 (**f**) cells (the green fluorescent cells) are in the S phase of mitosis. Representative images of DAPI staining in Ad-V- or Ad-TIPE2-infected EC9706 (**e**) and EC109 (**f**) cells (the blue fluorescent cells) represent all of the cells. Cell proliferation rates were also determined by EdU cell proliferation assay in Ad-V- or Ad-TIPE2- infected EC9706 (**g**) and EC109 (**h**) cells at the 3th day after infection, *P < 0.05

### TIPE2 overexpression inhibited cell invasion and induced apoptosis in esophageal carcinoma cells

Transwell invasion assay further demonstrated that adenovirus-mediated TIPE2 overexpression markedly repressed invasion capability of EC9706 (Fig. 3a) and EC109 (Fig. 3b) cells compared with Ad-V control group. Furthermore, we further validated that the enforced expression of TIPE2 strikingly induced apoptosis in EC9706 (Fig. 3c) and EC109 (Fig. 3d) cells compared with Ad-V control group, as illustrated by flow cytometry analysis. Taken together, our study proved that adenovirus-mediated TIPE2 overexpression inhibited invasion and facilitated apoptosis in esophageal carcinoma cells.

**Fig. 3:** TIPE2 overexpression suppressed invasion and induced apoptosis in esophageal carcinoma cells. Transwell assay was employed to assess invasion capability in Ad-V- or Ad-TIPE2-infected EC9706 (**a**) and EC109 (**b**) cells. Cell apoptosis rates were measured in Ad-V- or Ad-TIPE2-infected EC9706 (**c**) and EC109 (**d**) cells at the 3th day after infection, *P < 0.05

### TIPE2 overexpression inhibited tumor growth in esophageal carcinoma in vivo

Subsequently, to further explore the effect of TIPE2 on tumor growth in vivo, xenograft tumor models were established by injecting with EC9706 cells infected with Ad-V or Ad-TIPE2 cells into nude mice. As displayed in Fig. 4a, c, adenovirus-mediated TIPE2 overexpression strikingly hindered tumor growth, as evidenced by the reduced tumor volume (Fig. 4a) and tumor weight (Fig. 4c). H&E staining was used as a rough method to evaluate the effect of TIPE2 overexpression on tumor cell viability. PCNA has been identified as a critical mediator in DNA replication process [14]. Hence, PCNA as a proliferation marker was used to assess cell proliferation in Ad-V or Ad-TIPE2-infected xenograft tumor. As shown in Fig. 4b, adenovirus-mediated TIPE2 overexpression resulted in a marked decrease of PCNA expression in vivo compared with Ad-V control group, indicating TIPE2 inhibited the proliferation of esophageal carcinoma cells in vivo. Together, these data showed that TIPE2 overexpression inhibited tumor growth in vivo.

**Fig. 4:** TIPE2 overexpression inhibited tumor growth in vivo. Xenograft tumor models were established by injecting with EC9706 cells infected with Ad-V or Ad-TIPE2 into the flank region of nude mice. **a** The tumor volume was monitored every 3 days for 24 days. **b** Resected xenograft tumor tissues were processed to perform IHC assay and H&E staining. **c** The representative photographs of xenograft tumor tissues were obtained and the mean weight of resected xenograft tumors was measured at the 24th day after infection, *P < 0.05

### TIPE2 overexpression suppressed activation of the Wnt/β-catenin signaling pathway in vitro and in vivo

Previous studies showed that TIPE2 was closely associated with Wnt/β-catenin pathway in glioma [10]. Hence, the effect of TIPE2 on the Wnt/β-catenin pathway was further assessed in EC9706 cells and xenograft tumors infected with blank Ad-V adenovirus or Ad-TIPE2 adenovirus. The results manifested that adenovirus-mediated TIPE2 overexpression suppressed the expressions of β-catenin, c-Myc, cyclinD1 in Ad-TIPE2-infected EC9706 cells and xenograft tumors compared with Ad-V control group respectively in vitro (Fig. 5a) and in vivo (Fig. 5b). The results implied that adenovirus-mediated TIPE2 overexpression inhibited cell proliferation via suppressing activation of the Wnt/β-catenin signaling.

**Fig. 5:** TIPE2 overexpression suppressed activation of the Wnt/β-catenin signaling pathway in vitro and in vivo. **a** Western blot assay was performed to detect the expressions of β-catenin, c-Myc, and cyclinD1 in EC9706 cells infected with Ad-V or Ad-TIPE2 at the 3th day after infection. **b** β-catenin, c-Myc, and cyclinD1 expressions were also measured in Ad-V- or Ad-TIPE2-infected xenografts tumor tissues, *P < 0.05

## Discussion

TIPE2 is a member of tumor necrosis factor (TNF)-α-induced protein 8 (TNFAIP8) family, which also includes TNFAIP8, TIPE1 and TIPE3 members [6]. Previous studies showed that TNFAIP8 family was implicated in the development and progression of various cancers such as gastric adenocarcinoma and ovarian carcinoma [15, 16]. Moreover, TNFAIP8 family has been verified to be closely associated with clinicopathological characteristics and prognosis of esophageal carcinoma patients [17]. As mentioned above, TIPE2 has been identified as a tumor suppressor in multiple malignancies. For instance, it was reported that TIPE2 overexpression hampered proliferation, epithelial–mesenchymal transition (EMT) process, migration, as well as invasion in prostate carcinoma [11]. Additionally, enforced expression of TIPE2 was revealed to suppress cell proliferation, colony formation and invasion in lung carcinoma cells, and suppressed lung carcinoma tumor growth in vivo [9]. Notably, it was also manifested that TIPE2 suppressed activation of oncogenic gene Ras, indicating that TIPE2 played a critical role in the development of carcinoma [18]. The present study illustrated the roles and molecular mechanisms of TIPE2 in esophageal carcinoma.

Firstly, we demonstrated that TIPE2 expression was downregulated in esophageal carcinoma tissues and cells compared with normal counterparts, which was in accordance with the studies in other cancers such as non-small cell lung cancer [9]. Previous studies manifested that abnormal expression of TIPE2 was closely correlated with pathological processes of cancer including proliferation, migration, invasion and apoptosis [11, 19]. Furthermore, it was documented that adenovirus-mediated TIPE2 overexpression inhibited the growth of gastric cancer xenografted tumors [20]. Hence, we further investigated the effect of TIPE2 overexpression on the progression of esophageal carcinoma in vitro and in vivo. The results showed that adenovirus-directed TIPE2 overexpression strikingly suppressed proliferation and invasion, as well as induced apoptosis in esophageal carcinoma cells in vitro. In vivo assay further demonstrated that adenovirus-mediated TIPE2 overexpression markedly blocked tumor growth in xenograft tumors of esophageal carcinoma. Therefore, we concluded that TIPE2 acted as a tumor suppressor in the development and progression of esophageal carcinoma.

Subsequently, the molecular mechanism of TIPE2 was further explored in esophageal carcinoma. TIPE2 has been demonstrated to be closely correlated with the Wnt/β-catenin pathway in cancer. For instance, TIPE2 suppressed hypoxia-triggered the Wnt/β-catenin pathway activation in glioma [8]. Moreover, TIPE2 overexpression hampered metastasis by promoting β-catenin degradation and inhibiting β-catenin signaling pathway in gastric cancer [10]. In the present study, we demonstrated that adenovirus-mediated TIPE2 overexpression suppressed the expression of β-catenin in EC9706 cells and xenograft tumors of esophageal carcinoma, indicating that TIPE2 acted as a tumor suppressor by inactivating the Wnt/β-catenin pathway in esophageal carcinoma. β-catenin, a critical component of the Wnt signaling cascade, has been demonstrated to be implicated in the progression of various carcinomas including esophageal carcinoma [20–24]. For instance, depletion of β-catenin reversed HIF-1α-induced EMT process in human prostate carcinoma cells [25]. Additionally, β-catenin downregulation hindered proliferation of esophageal carcinoma cells [22, 26].

Moreover, β-catenin as a transcriptional activator can induce the transcription of multiple genes such as c-myc, cyclinD1, c-jun and survivin [27]. Wang et al. reported that β-catenin knockdown suppressed the expression of downstream effectors such as c-myc and cyclinD1 in esophageal carcinoma [28]. Additionally, the expressions of β-catenin and c-myc was closely correlated with invasion depth and lymph node metastasis together with prognosis of esophageal carcinoma [28, 29]. C-myc, a downstream effector of β-catenin, also has been demonstrated to be implicated in the development of various tumors including esophageal carcinoma [29–32]. Moreover, as a downstream effector of β-catenin, cyclinD1 has been identified as a vital mediator of cell cycle and cancer progression [33, 34]. In esophageal carcinoma, cyclinD1 suppression was associated with a decreased cell proliferation, a reduced tumorigenicity, as well as a good prognosis [35, 36]. CyclinD1 acted as an oncogene and was frequently overexpressed in esophageal carcinoma [37]. Hence, the effects of TIPE2 on expressions of c-myc and cyclinD1 in esophageal carcinoma were further explored. In accordance with these data, our results showed that adenovirus-mediated TIPE2 overexpression suppressed the expressions of c-myc and cyclinD1 in esophageal carcinoma in vitro and in vivo.

## Conclusions

In conclusion, our study demonstrated that TIPE2 expression was significantly decreased in esophageal carcinoma tissues and cells. Moreover, TIPE2 overexpression remarkably inhibited cell proliferation and tumorigenesis of esophageal carcinoma in vitro and in vivo. Mechanistic analysis manifested that TIPE2 exerted its anti-tumor effect by suppressing the Wnt/β-catenin pathway in esophageal carcinoma. Therefore, TIPE2 might be useful as a crucial prognostic biomarker and potential therapeutic target for esophageal carcinoma.

## Abbreviations

TIPE2: tumor necrosis factor-α-induced protein-8 like-2
PCNA: proliferating cell nuclear antigen
BSA: bovine serum albumin
HEEC: normal human esophageal epithelial cells
TNFAIP8: tumor necrosis factor (TNF)-α-induced protein 8
EMT: epithelial–mesenchymal transition
